# Effects of Acupuncture and Rehabilitation Training on Limb Movement and Living Ability of Patients with Hemiplegia after Stroke

This article has been retracted.

**DOI:** 10.1155/2022/2032093

**Published:** 2022-04-26

**Authors:** Juhua Zhang, Yingmei Mu, Yunxia Zhang

**Affiliations:** Neurosurgery, Shandong Yuhuangding Hospital, Yantai, 264000 Shandong, China

## Abstract

Stroke is a disease with a high disability rate, having a serious impact on that patient's working and daily survival quality and bringing economic burden to the family and society. Patients with stroke hemiplegia are mostly tetraplegic and have difficulty regulating their balance, and their long-term symmetry has been destroyed. The application in the rehabilitation process of acupuncture in patients with hemorrhagic stroke may produce unexpected effects. It is very effective to study the effect of acupuncture combined with rehabilitation training on limb movement and patient survival. It is very helpful in improving normal motor function and normal life, increasing joint mobility and muscle strength, and reducing muscle tension. In this paper, it is found that the observational group has a complication rate of 2.13%, in contrast to 17.02% as in the group of control, and the pin-prick combined with a rehabilitative training makes a significant improvement to the patients. This study provides suggestions for the study to investigate acupuncture combined with recovery exercise on limb movement and living capacities of people with stroke paraparesis.

## 1. Introduction

Acupuncture is a rehabilitation treatment for acute cerebrovascular diseases in recent years. It achieves the goal of “Internal Diseases and External Treatments,” by stimulating the meridian, promoting blood circulation and eliminating veins in the blood, and fully providing local and comprehensive treatment. At present, scalp acupuncture and hemispherical acupuncture are common in clinical treatment. Traditional Chinese medical theory believes that the head is where the IQ and the meridian merge. Through scalp acupuncture, IQ is adjusted to improve local microcirculation and increase brain blood. Cerebral edema flow and relief using different acupuncture points and different stimulating forces can lead to brain cell stimulation or inhibition of two-way regulation, stimulating the central dynamic nervous system, improving the signal input to the dynamic area of the cerebral cortex, and thereby promoting recovery.

Because the central nervous system is damaged, the patient's dynamic function is also reduced. If the patient does not receive systematic rehabilitation training, it will have serious consequences, which will greatly reduce the quality of life and put more burden on the patient's family. According to related research, when the central nervous cells of the human body are damaged, their adjacent brain cells are stimulated, and a part of their damaged nerve functions is distinguished and compensated. Control patients benefited from standard therapy only, with associated medications to restore neurological function in the patients. In contrast, it was found that acupuncture integrated with rehabilitation traveled far and above conventional therapy.

The Hachisuka A. et al. study found that pituitary stroke is usually the result of a hemorrhagic infarction of pituitary adenomas. Clinical manifestations are diverse, including asymptomatic cases, typical pituitary stroke, and even sudden death. Cerebral ischemia caused by pituitary stroke is very rare. It may be caused by vasospasm or tumor directly compressing the cerebral blood vessels [1]. The Satyarthee and Sharma study found the diagnostic value of DD and coagulation indicators for stroke, providing clinical basis for diagnosis (40 cases) and hemorrhagic stroke group (observation group 2, 20 cases), using a coagulometer to detect DD, PT, APTT, FIB, and AT-III. The results of Satyarthee and Sharma showed significantly higher levels of DD and FIB compared to the development of the controlled group (*p* < 0.01). In the observation subjects 1 and 2, the levels were significantly higher, APTT was significantly prolonged, and AT-III was significantly lower, with striking statistically significant differences (*p* < 0.05). Detecting indicators 1 and 2 were not significantly different (*p* < 0.05), and APTT and FIB were positively correlated with stroke (*r* = 0.422, 0.138, 0.171, *p* 0.05) [2].

Acquisitions of comorbid rehabilitation training combined with acupuncture can often have unexpected effects on limb movements and life skills in stroke patients with hemiplegia. In this paper, 94 stroke patients admitted from December 2019 to January 2020 were selected and compared with the reference. The rehabilitation status of the two groups of patients who received “acupuncture incorporating rehabilitation training and no acupuncture combing training” was observed. A better recovery effect with the combination of acupuncture and moxibustion training was observed than that without the combination of needle and moxibustion training. However, these studies still need to be more improved in experiments, especially to pay attention to the innovation of experimental methods.

## 2. Proposed Method

### 2.1. Acupuncture

It is the general term for acupuncture and exercise. With guidance from Chinese medical theory, moxibustion refers to the insertion of needles (often called pins) into a specific angle into a patient's torso. Particular areas will be stimulated to achieve a disease treatment goal. This puncture point is known as a point on the body and is called an acupuncture point. The most current acupuncture manual numbers 361 acupuncture spots throughout the entire body. It is done by rubbing or kneading, fumigation, ironing, and the application of heat stimulation to a “point” on the upper surface of the body to prevent and treat disease. There are also other methods such as moxibustion, moxibustion, core moxibustion, and mature moxibustion. In addition, there are other methods such a moxibustion, osier moxibustion, core moxibustion, and mature moxibustion. It includes “moxibustion” and “moxibustion with medicine,” as an important part of Oriental medicine, including acupuncture theory, the points, acupuncture techniques, and related equipment. During its formation, application, and preparation, the unique Chinese culture and regional characteristics are the result of the valuable heritage of Chinese cultural and social traditions, and in 2006, the school of Chinese medicine announced with the State Council that acupuncture was included in the first inscription of national intake of intangible cultural property [3, 4]. Therefore, there is also more and more clinical research on acupuncture.

In China, acupuncture can be used as a unique treatment for diseases. It is a medicine for internal and external treatment. Which is accomplished by guiding meridians and acupoints and applying certain methods to treat systemic diseases. Acupuncture is used to diagnose the causes of TCM and identify the methods that belong to nature, meridians, and injured organs according to the TCM practice and confirmed as belonging to the TCM category. Discussions are followed by respective prescriptions for acute treatment. Through the channeling of meridians and the regulation of hemoplasm, the functions of yin and yang are rendered relatively balanced for the preventing of diseases. It is part of the ancestral medical heritage and a unique and ethnic Chinese medical approach. Over the centuries, it has made outstanding contributions to the protection of national well-being and reproduction. It remains his task up until now and has won the popular trust [5].

The function of the meridian is to keep the meridian unblocked and exercise its normal physiological functions. This is the most basic and direct treatment method of acupuncture [6]. The meridian is the internal organs of the viscera and external limbs, and Qi and blood surgery are one of its main physiological functions. The meridian is not connected, the blood is not connected, and the clinical manifestations are pain, deafness, swelling, eczema, and other symptoms. Acupuncture chooses appropriate acupuncture methods and triangle needles to keep the meridians free and qi and blood normal [7].

### 2.2. Stroke Rehabilitation Training

#### 2.2.1. Guidance on Training Essentials

1. Provide good psychological care for patients and their families: patients and their families should be patiently informed about the purpose, methods, effects, and training of medical physical rehabilitation before rehabilitation training. Rehabilitation cannot be replaced by drugs. Only through early training can the remaining functions be restored in accordance with the “progressive” rehabilitation training plan and cannot be rushed. Only with the active participation of patients and the strong support of family members can rehabilitation training be successfully completed [2, 8, 9]
2. Maintain the correct position of good limbs: good limbs are not the same as functional limbs. This is a temporary location, designed from a therapeutic perspective. Most of the affected limbs in the acute phase of hemiplegia are now relaxed. Not only can it not move, but it can also lead to subluxation of the joints and damage to the soft tissues around the joints and even contracture due to abnormal posture for a long time. Good limb placement can play a role in inhibiting spasm patterns, preventing shoulder bruises and early separation movements. Play is an important measure to prevent many complications and improve rehabilitation [10, 11]

#### 2.2.2. Training Method

1. Posterior method: place your head on the pillow, tilt it slightly to the healthy side, refer to the affected side, the height of the pillow should be sufficient, and the thoracic spine should not be bent. Place a cushion below the patient's hip to move the affected pelvis forward to prevent hip flexion and external rotation. Place a small pillow under the patient's shoulder joint to push the scapula forward. Stretch your upper elbows on your pillow, and stretch your wrists backwards and your fingers. Place a sandbag on the outside of the thigh and the middle of the thigh to prevent hip dislocation and external rotation and a small pillow in the sleeping area to prevent knee joint extension
2. The lateral position below the affected side: the affected side's shoulder belt stretches forward, shoulder reflexes, elbows straight, wrists straight, and fingers straight. The affected limb is straightened, and the knee joint is slightly bent. The hips and knees of the lower limbs on the healthy side are bent, and a cushion is placed below to prevent the affected lower limbs from being squeezed together. A pillow is pressed against the back, and the upper body can be leaned on to obtain a relaxed posture [12, 13]
3. Above the affected side: the upper limb of the affected side is extended forward, and the shoulder joint is bent about 90 degrees. The floor is supported by cushions, and the healthy upper limbs can be placed freely. Hip and knee joints of the affected lower limbs are bent and placed on a cushion. The left hip is stretched, the knees are slightly bent, and the back is pressed against the pillow to relax the trunk. In order to prevent joint contraction and to maintain pressure in a specific position for too long, you must change the position in time according to the situation and generally reverse it every two hours. When changing positions, special care should be taken to protect the shoulder joints and do not pull the affected joints to prevent shoulder injuries [14–16]

#### 2.2.3. Problems to Pay Attention to during Training

1. Avoid intravenous amputation where possible: some patients and family members believe that the affected limb will not move this way, or that it is an intravenous infusion. I do not know that a healthy limb is free, but it does bring the repair of a damaged limb. Side effect. Due to insufficient blood return of the affected limb, coupled with sweating and limited movement, it is easy to cause hand swelling and tissue adhesion, increase the risk of shoulder-hand syndrome, and provide guidance and cooperation for rehabilitation nursing staff to facilitate patient limb repair [17, 18]
2. Academic practice should be avoided in limb rehabilitation training: limb paralysis is a common symptom of stroke patients, and joint training for the ability of amputated limbs is an important rehabilitation measure. The principle is to train in pain, and rehabilitation nurses must have stable knowledge in various fields such as neuroscience, anatomy, psychology, and medicine. Restore. On this basis, they should be processed manually to prevent rough handling. For patients with pain, you can take hot packs or painkillers before training to avoid shoulder dislocation, shoulder joint syndrome, and epilepsy during exercise; exercise should be slow and rhythmic, and the patient should be clearly explained before training. The purpose, content, function, and correct action items of the action inform the patient of the active part, direction, and regular muscles, and then, slowly perform passive activities 2-3 times so that the patient can feel the movement and gradually decrease in this case. Auxiliary active exercise volume [19, 20]
3. Pay attention to the scale and intensity of training during physical rehabilitation: patients often feel anxious when freely moving. Excessive exercise can cause modern compensatory exercise or pain and fatigue, which increases spasm and affects exercise results. Rehabilitation nurses should explain to patients and their families different training methods used at different rehabilitation stages, as well as monitor the general situation of patients, follow small- and long-term nursing principles, and gradually increase education, that is, to complete the total training and avoid the negative effects of overtraining from overtraining. Each time you train an action, you must maintain a precise attitude and focus your brain's thoughts on this action and the main part of your training body to “control” this behavior of the brain. Power is always a passive activity and cannot achieve the purpose of education. Training the passive activity in one's own active action is the real problem of training [21, 22]
4. Attention to the systemic and follow-up of rehabilitation training: to achieve a good training effect and in order to achieve the expected purpose of restoring physical function, it is necessary to carry out serious training at the prescribed time in accordance with the established plan. Classes and holidays should be avoided. Interrupted training is interrupted because the trainee cannot experience specific repetitive stimuli, cannot produce adaptive responses, and has no value to avoid focusing on any training. Although these sections ignore other sections, they must fully consider different joints, muscles, and different functions. Therefore, the restoration of limb function requires some persistence and family supervision
5. When performing physical rehabilitation training, care should be taken to avoid premature walking: some patients and their families are concerned about the slight mobility of the affected limbs. They want to achieve this. They cannot wait for intensive education of many people. Hold on and hold your hand to walk or climb the stairs. It is necessary to know that “not enough speed” does not focus on the training of basic movements and ignore the stages of the patient's movement pattern
6. Be careful when dealing with recovery after rejection: some patients become sensitive and vulnerable after illness, overreliance on doctors and their families, lack of initiative in rehabilitation education, and think that the doctor's technology is the treatment of fact. In effect, active training is much better than passive training [23]. Some failures tend to last longer and some even last a lifetime. Therefore, we should not only be interested in the training of patient care, we should pay attention to education or social education after the patients are repatriated, and fully guide family members to teach patients the knowledge and skills to maintain health and daily life. The patients have recovered to a good society and family status. After refusing treatment, the rehabilitation nurse must conduct a telephone return visit to understand the patient's self-service ability and training home guidance after treatment [24]

### 2.3. Application of Acupuncture in Stroke

Heme is the main manifestation of limb dysfunction in stroke patients, and the main reason is the neuron damage and transplantation abnormality. An implant includes impaired coordination between muscle groups, increased muscle tone, and limited joint mobility. Since joint motion is controlled by the contraction and relaxation of related muscle groups, joint mobility can be improved by strengthening the function of related muscle groups. Traditional Chinese medicine can promote local muscle blood circulation and alleviate the symptoms of edema and pain while improving muscle and neurotrophy, eliminate the pressure of neuroedema, and achieve the effects of promoting functional recovery and inhibiting muscle atrophy. The damage of the upper motor neurons prevents the release of the retroreflector in the lower center, which is the cause of hemophilic contraction, but the effect of simply applying traditional Chinese medicine to repair the damaged neurons is average. Acupuncture can select the puncture site according to the anatomy of the patient's limbs or muscles, stimulate nerve muscles, correct excitement imbalance and inhibit nerves, and promote nerve recovery. Medical aspects. Acupuncture can promote the movement of the affected limb, use and regulate the body's reflexes, strengthen central stimulation, and improve coordinated control of the affected limb. Limited joint mobility is a common manifestation of dyskinesia. Improving joint mobility is the main purpose of rehabilitation for semidisabled patients. Hip and knee joints are important joints that control the movement of the lower limbs, and it is not necessary to increase the effect of Chinese medicine on joint mobility. Muscle failure is the leading cause of stiff limbs. The enhancement of muscle strength after acupuncture combined with Chinese medicine is related to the improvement of muscle strength and the reconstruction of acupuncture function. In addition, the reduction of muscle tension after acupuncture with Chinese medicine is also the basis for increasing joint mobility.

## 3. Experiments

### 3.1. Materials and Methods

(1) General information: from December 2019 to January 2020, 94 stroke patients were selected and treated. Inclusion criteria are as follows: all patients met the diagnostic criteria in the 2016 American Heart Association/American Heart Association Brain Repair Guidelines. Depressive symptoms, signed informed consent, agreed to receive research training, no surgery or thrombolytic therapy, all patients appeared for the first time, and the course of disease was less than two weeks
(2) There was an observation group and a control group divided into 47 cases in each group by the contact ball method. The observer group had 26 cases of males and 21 cases of females, aged 54-76 years, meaning 65.2-1.4 years, including 23 cases of mongrel, 24 cases of right hemizygous, and 25 cases of male. The control group consisted of 22 females and 55 females, ~76 years old, mean age 65.3~1.3) years old, in which 24 cases of left hematoma and 23 cases of right hematoma
  1. First of all, it is necessary to correctly position and transform the limbs, try to keep the limbs in an anatomical functional position, and often move the limbs to prevent the pressure of ulcers
  2. Active and passive movements on the bed, such as upper arm abduction, elbow extension, lower limb extension, and back twist of knees and ankles
  3. To perform a certain massage repair, it is necessary to regularly massage the affected joints and muscles of the patient to accelerate the blood circulation of the limbs. Seated training
  4. Continuous balance training
  5. Stairs for walking and climbing
  6. Life skills training (including food, laundry, dressing, etc.)
  7. Resistance training: the above active and passive exercises are trained once a day in the morning. The total training time is 2~3 h/d for a total of 3 months. During the training, the patient can endure without feeling tired
  8. Get some psychological treatment
(2) Both groups of patients received conventional neurological treatment, and the nurses evaluated the patient's symptoms, combined with the cause to give the patient general treatment, assisted to actively fight the disease, and established a correct and good treatment mentality; the observation group was supplemented with rehabilitation training interventions. The specific content is as follows: the medical staff sets up a rehabilitation training intervention group consisting of the attending doctor, rehabilitation physician, and nurse and conducts training work around the content of rehabilitation training to actively improve its self-cognition level and comprehensive ability and develop rehabilitation training based on the patient's condition and actual situation. The plan mainly includes correct posture placement, changes, active and passive joint activities, early seated adaptive training, stance changes, and body center of gravity shifts and monitoring the patient's quality of life and mental state throughout the process. For patients with sexual psychology, the nurses carry out health training work around them in a timely manner, inform the patients of stroke, depression, treatment, and prognosis, improve the patient's self-cognition level, and enable them to actively cooperate with treatment and nursing work to ensure intervention effect. Acupuncture treatment was given, and patients were instructed to take the supine position and take acupuncture points such as Sanyinjiao, Shenmen, Sishencong, and Baihui to get Qi for 30 min, 1 time/d, with 10 d as a course of treatment; for patients with liver qi stagnation, Taichong and Hegu points can be added; those with phlegm fever can be added to the inner court and Fenglong acupoints, and the liver and fire are strong, and those with yin deficiency can be added with acupuncture points such as Taichong, Yongquan, and Taixi. Acupoint, rest 3 d after the end of the treatment course, and proceed to the next course according to the actual situation of the patient. Treatment group rehabilitation content: in addition to the same rehabilitation training as the control group, acupuncture was also used for functional rehabilitation. Acupuncture is mainly based on acupuncture points of the large intestine and stomach, supplemented by acupoints of the bladder and bile. At the beginning of the disease, only the affected side is punctured. After a long course of disease, the healthy side can be punctured first, and then, the affected side can be punctured. Mainly take ring jump, Yanglingquan, Zusanli, and Kunlun, and can take turns to Fengshi, Juegu, Yaoyangguan and other points. Acupuncture points with symptoms: Taiyang and Taichong with liver yang and hyperthyroidism; Fenglong and Hegu with wind and phlegm resistance; varus correction with foot inversion and Qiuxu through the sea; valgus with Zhongfeng, Taixi, and correction of eversion; foot droop with Jiexi and Taichong; and constipation with Fenglong and ditch. Acupoints and needles are routinely disinfected. In the acute phase, twist and diarrhea was used, and the needle was continuously applied for 10-15 minutes. During the recovery period, the needle was used for 20-30 minutes, and moxibustion was performed on the acupuncture points. Once a day, 10 d is a course of treatment, rest 3 d, and continue treatment

### 3.2. Research Indicators

Observe the effects after the intervention, including the occurrence of complications, neurological deficit scores, mental health scores, and changes in depression scores before and after the intervention. The NIHSS scoring system was used to assess the degree of neurological deficits. The score was 100 points. The smaller the score, the smaller the neurological deficit, and vice versa. The SCL-90 symptom self-assessment scale was used to assess the mental health of patients. The scale items are as follows: thinking, living habits, consciousness, interpersonal relationships, emotions, feelings, behaviors, diet and sleep, etc., from none, very light, medium, biased, and severely corresponding 1 to 5 grades; scale score is 450 points; the lower the score, the better the mental health. The psychiatric class A PHQ-9 score was used to assess depression, and the questionnaire survey was used. The normal score was 0 to 4 points, with depressive symptoms; 5 to 9 points, the obvious depressive symptoms; and 10 to 14 points, severe depressive symptoms: 15~27 minutes. Efficacy criteria are as follows: Barthel index of daily living ability, FAC lower limb walking function score, Fugl-Meyer score, and other treatment effects were evaluated. The statistical data of the statistical method was expressed as *z* ± 5.

### 3.3. Data Processing

Data processing was performed using the statistical software SPSS21.0. The calculation data was described by *x* ± *s* and *t* test; count data was expressed by rate and *χ*^2^ test; *α* =0.05 was used as the test criterion. The entire data processing process is shown in Figure 1.

## 4. Discussion

### 4.1. Control Group

Higher levels of complications in the two groups are presented in Table 1.

Table 1 shows that the complication rate in both groups was 2.13% (1/47) compared against the observation group, being 17.02% (8/47) lower than that in the control group, for which the variation was of statistical relevance (*p* = 0.035).

The score of neurological deficits and mental health ratings of the two groups is compared in Table 2.

As seen in Table 2, the neurological deficit rating and mental health score in both groups with statistically significant differences (*p* < 0.05) were lower on the control group.

Comparison of before and after interventions for both groups is shown in Table 3.

The depression scores of the two groups before and after the intervention were compared according to Table 3. With the observation group, depression scores were lower when compared to the control group after the intervention, and differences were observed which was statistically important (*p* < 0.05).

From Tables 1–3 before and after the comparison, we can know that poststroke depression is one of the common sequelae of patients with clinical stroke, and the incidence is 31.2%~63.1%, which is at a very high level. After the occurrence of depression sequelae, the patient's mental state is in a deep and depressed state for a long time, and he loses attention to life. Some severely depressed people may even ignore life and give up life, which seriously affects their prognosis and health. Moreover, in the clinic, most patients with stroke have language dysfunction, which makes it impossible to detect the depressive symptoms in time, so it is necessary to strengthen the observation of patients' mental and emotional states. Rehabilitation training intervention is a clinical intervention measure applied in recent years. It mainly implements interventions for patients with limb dysfunction, evaluates their limbs and emotions early, and implements guidance based on their characteristics to promote their limb function recovery as soon as possible. The results showed that in the observation group, the risk of complications after rehabilitation intervention was effectively reduced. After the intervention, the patients' neurological function and psychology and depression scores were in a good range, which further confirmed the significant effect of rehabilitation intervention in clinical. The clinical application of rehabilitation training in poststroke depression patients helps to alleviate and enlighten the patient's negative psychology and adverse emotions, enabling them to face treatment and rehabilitation training with a good attitude and to maximize their impact on the disease. Implementing acupuncture interventions can effectively improve the patient's own tolerance, improve their physical condition through dredging channels and channels, and promote the improvement of the intervention effect.

Table 4 shows the Barthel index of the two groups after rehabilitation.

This is seen in Table 4, the Barthel index was significantly higher in both groups after rehabilitation than before rehabilitation, and the difference was dramatically significant (*p* < 0.05). It also shows that the Barthel index of the control group was higher than that of the treatment group on rehabilitation, and there was a significant difference (*p* < 0.05).

### 4.2. Comparison of FAC and Fugl-Meyer Scores

The FAC and Fugl-Meyer lower limb basic motor function scores of the two groups of patients after rehabilitation are shown in Figure 2.

As seen in Figure 2, the FAC results after recovery were significantly higher than those before recovery in both groups, with a remarkable variance (*p* < 0.01). After recovery, the FAC scores in the treatment oriented group were significantly higher from the control group (*p* < 0.05). It can also be seen from Figure 1 that the degree of basic motor function of Fugl-Meyer's lower limbs was significantly higher after rehabilitation than before rehabilitation (*p* < 0.01). For the basic motor function score, difference was significantly more than control group (*p* < 0.05).

Acupuncture and rehabilitation both advocate early treatment, and early patient position care is the main link of limb rehabilitation. Acupuncture or modern rehabilitation treatment as soon as possible after the vital signs of stroke patients are stable can effectively improve the symptoms of motor function and neurological deficits and improve their daily activities.  Figure 3 is a comparison of FAC's lower limb walking function score.

The lower extremity FAC score is an evaluation of the lower limb walking ability of a half-life patient, and the Fugl-Meyer score is an assessment of the underlying dynamics of surgical treatment of the lower extremity of a hemiplegia patient.  Figure 3 shows that the results of rehabilitation training in the two groups of patients are significantly higher than before, indicating that there is a significant difference between before rehabilitation and before acupuncture, and that traditional rehabilitation methods and acupuncture have a certain rehabilitation effect. According to the literature, acupuncture can stimulate the excitement of motor neurons, promote the formation of new high-level centers and peripheral transportation routes, and mutually promote rehabilitation training. However, it can be seen from Figure 2 that the FAC and Fugl-Meyer scores of the treatment group are significantly higher than those of the control group, and it shows that acupuncture combined with traditional repair methods has a better ability to recover walking. For a long time, traditional recognition in the field of neurological interventions considered spasm to be the most important factor limiting motor function recovery. Treatment strategies focus on normalizing muscle tone and promoting the formation of normal forms of exercise. Patients with hemiplegia are predominantly spasm of the sixth muscle of the knee, which leads to irregular bending of the knee joint. Acupuncture is mainly based on acupuncture points near the muscles of the affected limbs, which can reduce reflex tension and muscle tension. Combined with techniques that promote confrontation and nerves in rehabilitation training, it can improve the motor function of the affected limb and the overall physical performance of the body. It is not necessary to have a promotion effect similar to or better than promotion. Acupuncture stimulates active muscles, which is basically a regional sensory input that can stimulate motor neurons, stimulate the production and strengthening of muscle tension, and stimulate motor neurons to promote traffic shunting.

The effective rates of the treatment group and control group are shown in Figure 4 and Table 5.

The clinical efficacy can be seen in Figure 4 and Table 5: according to the evaluation criteria, there was an overall effective rate of 97.5% in the treated group and 75.0% in the control group. It was better in the treatment group with a lower neurological deficit score after treatment than in the control group compared to the control group.

In the treatment group together with the controls, the limb motor function scores and daily living ability are shown in Figure 5.

As seen in Figure 5, the limb motor function scores and daily living ability in the treating group improve significantly compared to the control group, and the difference is statistically significant (*p* < 0.01) when comparing the two groups. There was a statistically significant difference compared with that before treatment (*p* < 0.01). In the treatment period, no adverse events and side effects occurred. There was no significant change in heart rate and blood pressure before and after treatment in the treatment group. The rehabilitation of patients with stroke hemiplegia can be divided into different stages (including soft paralysis, spasticity, and recovery), and the different acupuncture treatments at different stages are satisfactory.

The difference between FMA-L and MWS before and after treatment in the two groups is shown in Figure 6.

As seen in Figure 6, the differences in FMA-L and MWS before and after treatment in both groups were not significant (*p* > 0.05) compared to FMA.L and MWS for both groups before treatment. There were elevated FMA-L and MWS in both groups after treatment, but the differences were statistically significant (*p* < 0.05). Both indices were higher than the control group after of the treatment, and the difference was statistically significant (*p* < 0.01). Time-dependent parameters of gait of the two groups before and after treatment were compared. There was an increase in gait frequency, stride length, affected and habilitation side stride length, gait cycle, and leg bolstering time after treatment, and the differences were statistically significant (*p* < 0.05). Each indicator was better than the core group with statistically meaningful differences after treatment (*p* < 0.05).

## 5. Conclusions

Stroke is a common disease in clinical neurology. It is mainly caused by the sudden rupture or blockage of blood vessels in the brain. After the illness, patients may experience dizziness, numbness, vomiting, and hemiplegia. In some severe cases, neurological and motor functions may be impaired, which may threaten their normal life and health. Acupuncture combined with rehabilitation training is effective in treating poststroke interventions. It can improve patients' mental state, depression, and neurological function and effectively reduce the impact of other complications on their prognosis.

This article uses a comparative experiment to compare acupuncture and rehabilitation training in patients with stroke. The first group did not use acupuncture combined with rehabilitation training, with the last group which employed acupuncture combined with restoration training, which was found to improve muscle strength. Limb function improves balance and coordination between muscle groups. During recovery, convulsions in the affected limb were relieved. This treatment is mainly based on acupuncture and antidiarrhea, which is beneficial to improve blood circulation in the extremities, increase tissue stimulation, and gradually recover from separated, thin, and controllable surgery, which significantly improves the patient's limb function and daily life. Therefore, the flexible use of acupuncture at different stages in patients with hemistroke is beneficial to functional recovery.

This article establishes comparative experiments and shows that a large number of patient rehabilitation training data show that acupuncture has a great effect on the rehabilitation training of stroke patients. The research in this article is limited to the analysis of clinical manifestations and prognosis of patients, and the mechanism of its impact is not clear. Therefore, it is still necessary to conduct analysis and research around the core theories of this study in order to contribute to the further improvement of clinical intervention. This article studies the effects of acupuncture combined with rehabilitation training on the physical activity and living capacity of stroke patients with hemiplegia.

This study found that lower limb motor operation, walking ability, and daily life in the observation group were significantly improved, and acupuncture combined with rehabilitation training significantly improved limb motion and survival evidence for stroke patients and intermission. Acupuncture can promote the movement of the affected limb, utilize and regulate the body's reflexes, strengthen central stimulation, and strengthen coordinated control of the affected limb. In combination with rehabilitation for improved limb circulation and limb survival, needles can have an improving action on stroke and hemiplegic patients. We studied the effect of acupuncture combined with convalescent training on limb movement and living capacity in stroke hemiplegic patients. This paper provides guidance for the study of needles combined with rehabilitation training on limb motion and living capabilities in stroke patients with paraplegia.

## Figures and Tables

**Figure 1:** Data processing process.

**Figure 2:** Comparison of FAC and Fugl-Meyer scores.

**Figure 3:** Comparative analysis of FAC and Fugl-Meyer before and after rehabilitation.

**Figure 4:** Comparison of total effective rate between the two groups (example).

**Figure 5:** Comparison of the functions of the two groups before and after treatment (x ± s, n = 20).

**Figure 6:** Comparison of FMA-Ll and MWS between the two groups before and after treatment (*x* ± *s*).

**Table 1:** Comparison of the incidence of complications between the two groups (*n*).

Group	Number of cases	Intracranial hypertension	Glycemic change	Pneumonia	Total incidence (%)
Observation group	47	1	0	0	2.13%
Control group	47	3	3	2	17.02%
*X* ^2^ value	0	0	0	0	4.424%
*p* value	0	0	0	0	0.035%

**Table 2:** Comparison of neurological deficit score and mental health score between the two groups (*x* ± *s*).

Group	Number of cases	Neurological deficit score	Mental health score
Observation group	47	2.36 ± 0.26	36.65 ± 2.32
Control group	47	4.56 ± 0.22	78.25 ± 1.98
*t* value		44.284	93.505
*p* value		<0.05	<0.05

**Table 3:** Comparison of depression scores between the two groups before and after intervention (*x* ± *s*).

Group	Number of cases	Before intervention	Prognosis after intervention	t value	*p* value
Observation group	47	14.65 ± 3.21	3.20 ± 0.13	24.434	>0.05
Control group	47	14.66 ± 3.22	6.625 ± 0.25	17.066	<0.05
*t* value		0.015	83.205		
*p* value		>0.05	<0.05		

**Table 4:** Comparison of Barthel index in daily living ability.

Group	*n*	Before rehabilitation	After rehabilitation
Treatment group	30	25.12 ± 9.13	65.41 ± 13.55
Control group	30	22.83 ± 8.32	42.24 ± 12.08

**Table 5:** NIHSS scores of the two groups before and after treatment.

Group	Reciprocal	Before treatment	After treatment
Treatment group	40	28.53 ± 6.2	11.12 ± 0.25
Control group	40	28.64 ± 5.5	19.5 ± 3.25
P		>0.05	<0.05

## Data Availability

No data were used to support this study.
